# Monitoring Cardiovascular Problems in Heart Patients Using Machine Learning

This article has been retracted.

**DOI:** 10.1155/2023/9738123

**Published:** 2023-02-08

**Authors:** Ahmed Al Ahdal, Manik Rakhra, Rahul R. Rajendran, Farrukh Arslan, Moaiad Ahmad Khder, Binit Patel, Balaji Ramkumar Rajagopal, Rituraj Jain

**Affiliations:** ^1^Department of Computer Science Engineering, Lovely Professional University, Jalandhar, Phagwara, Punjab, India; ^2^Department of Mechanical Engineering and Mechanics, Lehigh University, Bethlehem, Pennsylvania, USA; ^3^School of Electrical and Computer Engineering, Purdue University, West Lafayette, Indiana, USA; ^4^Department of Computer Science, Applied Science University, Eker, Bahrain; ^5^Indukaka Ipcowala Institute of Management, Charotar University of Science and Technology (CHARUSAT), Changa, Gujarat, India; ^6^Cognizant Technology Solutions, Chennai, Tamil Nadu, India; ^7^Department of Electrical and Computer Engineering, Wollega University, Nekemte, Ethiopia

## Abstract

The World Health Organization reports that heart disease is the most common cause of death globally, accounting for 17.9 million fatalities annually. The fundamentals of a cure, it is thought, are important symptoms and recognition of the illness. Traditional techniques are facing many challenges, ranging from delayed or unnecessary treatment to incorrect diagnoses, which can affect treatment progress, increase the bill, and give the disease more time to spread and harm the patient's body. Such errors could be avoided and minimized by employing ML and AI techniques. Many significant efforts have been made in recent years to increase computer-aided diagnosis and detection applications, which is a rapidly growing area of research. Machine learning algorithms are especially important in CAD, which is used to detect patterns in medical data sources and make nontrivial predictions to assist doctors and clinicians in making timely decisions. This study aims to develop multiple methods for machine learning using the UCI set of data based on individuals' medical attributes to aid in the early detection of cardiovascular disease. Various machine learning techniques are used to evaluate and review the results of the UCI machine learning heart disease dataset. The proposed algorithms had the highest accuracy, with the random forest classifier achieving 96.72% and the extreme gradient boost achieving 95.08%. This will assist the doctor in taking appropriate actions. The proposed technology will only be able to determine whether or not a person has a heart issue. The severity of heart disease cannot be determined using this method.

## 1. Introduction

Heart disease is the leading risk factor for death globally, taking 17.9 million lives each year. CVDs are a group of heart and blood vessel problems. The diagnosis of heart disease has been found to significantly reduce incidence and mortality in both known and unknown cardiovascular disease patients. The most significant personality-related lifestyle factors for cardiovascular attack and stroke are poor diet, insufficient physical activity, tobacco, and excessive drinking. Individuals' psychological behaviours may lead to hypertension, irregular blood sugar levels, increased plasma lipid levels, and overweight. Certain intermediate health conditions are detected in medical settings and are associated with increased cardiovascular risk, strokes, heart failure, and other issues. Young individuals are frequently affected by cardiovascular illnesses these days. So according to statistics and past experience, a heart attack, also known as a myocardial infarction, is frequently the leading cause of death in the United States. A heart attack occurs every 40 seconds in the United States. Because it impacts blood flow, stroke is classified as a heart disease. However, the cause of a stroke is not the heart but rather problems with blood supply to the brain. Ischemic strokes account for 87% of all strokes and are caused by blockages in the blood arteries that provide oxygen and blood to the brain. A heart arrhythmia is any abnormal cardiac rhythm, particularly one with an unpredictable pulse or speed. Without it, the heart does not operate properly.

The following are common examples of cardiovascular problems:

- Coronary heart disease: This occurs when blood circulation to the cardiac muscle is limited or stopped due to large levels of fat (atheroma) inside the coronary veins. An artery is a major blood vessel that transports blood to the heart [1]. When blood vessels narrow, leading to atheroma formation, blood flow to the heart muscle is reduced. This can cause angina (chest pains). A heart attack can occur if a coronary artery becomes completely blocked. This is a medical emergency that demands immediate attention. When the walls of the coronary arteries become too thin or cholesterol blockages form, this condition develops [2, 3]. Particularly during intense exertion, the heart may not receive enough oxygen-rich blood if these arteries close. It happens when a coronary artery's inner layer is wounded or destroyed. Fatty plaque deposits occur at the injury site as a result of this damage [4, 5].
- Peripheral arterial disease: This develops when the arteries feeding the limbs get clogged (usually the legs). Leg discomfort when walking is the most prevalent sign of peripheral arterial disease. This is usually felt in one or both knees, hips, and calves. Muscle pain, dull discomfort, or heaviness in the leg muscles are all possible symptoms [6]. It frequently comes and goes and is exacerbated by leg exercises such as walking or stair climbing. Peripheral arterial disease (PAD) is defined as the constriction or obstruction of the veins that carry blood from the heart to the legs. The major cause is the buildup of fatty plaque in the arteries, known as atherosclerosis [7, 8]. PAD can damage any blood artery; however, it more commonly affects the legs than the arms. Nonetheless, up to four out of ten people with PAD experience no leg pain. Walking may cause soreness, aches, or cramps in the pelvis, hip, thigh, or calf (claudication) [9, 10].
- Myocarditis: It is an inflammation of the inner muscles of the heart caused by a variety of parasitic and microbial infections. It is a rare illness with only a few symptoms such as joint discomfort, limb swelling, or fever that cannot be diagnosed from the inside. Myocarditis is uncommon, but when it does occur, it is typically caused by an interior infection. Infections with microorganisms, fungi, parasites, viruses (most often, viruses that cause the flu virus, influenza, or COVID-19), or any other microorganisms can induce myocardial inflammation. Autoimmune diseases such as lupus, sarcoidosis, and others can trigger myocarditis due to the immune system's ability to target any organ in the human body, along with the heart, and cause inflammation. Myocarditis can also be caused by drug usage, environmental exposure, or dangerous chemicals.
- Congenital heart disease: It is a condition that is associated with one or even more structural cardiovascular issues which have occurred since birth. A “congenital” handicap is one that is apparent at birth [11]. Congenital heart disease, commonly referred as congenital heart defect, changes the nature of blood through the heart from birth. Congenital heart abnormalities do not always cause symptoms. Complicated defects, on the other hand, could lead to life-threatening consequences. Infants with congenital cardiac disease can now live into adulthood because of breakthroughs in detection and therapy. Congenital heart disease symptoms may not develop until the patient is an adult.
- An arrhythmia is an irregular heartbeat: If a person has this condition, their heart may beat excessively rapid, extremely slow, very early, or in an irregular rhythm. This occurs when the electrical impulses that control heartbeats fail. An irregular heartbeat can feel like a rushing or fluttering heart.

Myocarditis is heart muscle inflammation (myocardium). The capacity of the heart to pump blood might be hampered by inflammation. Chest discomfort, shortness of breath, and fast or irregular heartbeats are all symptoms of myocarditis (arrhythmias). Myocarditis can be caused by any of the following factors:

*Viruses*. Many viruses have been linked to myocarditis, including adenovirus, COVID-19, hepatitis B and C, gastrointestinal infections (echoviruses), and HIV, the virus that causes AIDS. Bacteria that can cause myocarditis include staphylococcus, streptococcus, diphtheria, and Lyme disease bacteria.

*Parasites*. Trypanosoma cruzi and toxoplasma are two examples. Certain medications or illegal drugs and chemicals or radiation cause some cardiac arrhythmias, but most are relatively innocuous. Arrhythmias, just from the other hand, may cause significant, even deadly, symptoms and issues whether they are highly irregular or originate in a weak or wounded heart [12]. Heart arrhythmias, which can cause fluttering or racing, are typically harmless. Some cardiac arrhythmias, on the other hand, can be painful and even fatal. A person's heart might well be rapid or sluggish for a myriad of purposes [13, 14]. For example, the pulse may rise during exercise and fall during sleep. Medicines, catheter treatments, or fast, slow, or irregular heartbeats could be managed or eliminated through implanted devices or surgery. Heart attacks and strokes are triggered by a restriction in the flow of blood to the heart and brain, a lack of physical exercise, smoking cigarettes, and excessive drinking. People with relatively high blood pressure, moderately high blood glucose, and moderately high blood lipids are more vulnerable, as well as those who are overweight or obese, may experience specific effects as a result of their health behaviours. Primary data may be used to assess these “intermediate risk variables.” Typically, no signs of blood vessel disease are noticed. A stroke or heart attack might be the initial indication of a disease. Pain and swelling in the arms, shoulders, or elbows. Furthermore which generally is fairly significant, the person may experience difficulties breathing or get breathless, nausea or vomiting, light-headedness, cold sweats, and pallor. Individuals diagnosed with heart disease, which is more common in women than in men, should have access to appropriate equipment and treatment. 1- Aspirin, 2- beta blockers, 3- angiotensin converting enzyme inhibitors, and 4- statins are all necessary medications that should be taken [15, 16].

### 1.1. Contributions

1. A comprehensive analysis was carried out to investigate various existing machine learning algorithm techniques and methods that were used in the predication of heart diseases. Scanning, visualizing, and monitoring of patients were also done.
2. Several machine learning techniques and strategies have already been contrasted and categorized based on their traits, efficacy, and effectiveness. This article proposes a new method for predicting heart disease with the highest accuracy of 96.72%.

### 1.2. Machine Learning History

This section discusses the history of machine learning in the medical field for last 20 years, from 2000 to 2020.

Figure 1 shows the history of machine learning in healthcare, starting with Joseph Weizenbaum who first introduced Eliza in 1964. Eliza was capable of having chat communication through implementing natural language processing approach-based matching and replacement techniques to mimic human speaking, setting the framework for future ChatterBots. And this was considered as the golden year of artificial intelligence; the release of the first computer-based medical research tool in 1975, accompanied by the NIH's initial annual AIM conference, highlighted the importance of artificial intelligence in the medical area. The scope of machine learning in healthcare has expanded with the discovery of deep learning in the 2000s and the publication of DeepQA in 2007. Furthermore, for the first time, CAD was used in endoscopy in 2010, and the first PharmBot was founded in 2015. In 2017, the Food and Drug Administration approved the first cloud-based deep learning application, marking the beginning of the use of artificial intelligence in healthcare. Numerous AI experiments in gastroenterology were conducted between 2018 and 2020.

### 1.3. ML Application on Healthcare

A massive data report and clinical diagnosis of the patient's cure and treatment are extremely difficult to set up in an accurate way; otherwise, these will be affected due to insufficient storage or management. This amount of data needs special means or tools to extract and process efficiently, by using one of the machine learning applications such as a classifier which can divide the data according to their attributes; this can be used in medical data analysis or disease detection [17]. ML was initially designed to observe medical data sets. In the last few years, ML technologies have achieved great work regarding diagnostic disease. Many reports and records from different modern hospitals have shown the efficiency of ML technologies' results. Machine learning has come a long way since the days when it provided voice recognition, rapid online search, and self-driving vehicles. Today it is present everywhere and can be used several times each day. In the medical field, it is used in various disciplines such as drug discovery, helps in complex surgeries to assist surgeons, and provides an electronic health record (HER), which is an alternate opinion for prediction. Several industries are implementing machine learning, and healthcare can indeed be one of their priority works such as Stanford, which is employing a machine learning technique developed by Google to detect cancer, specifically skin cancer. Machine learning is referred to as “training” by experts, and the outcome is referred to as a “model.” The model is fed input, and it generates new knowledge based on what it has already learned.  Figure 2 shows different machine learning applications in the healthcare sector which are as follows:

- *Identification of Diseases and Diagnosis*. For example, QuantX is a machine learning application and artificial intelligence are at the core of it. It addresses patients' and clinic administrators' essential needs and delivers information to assist in faster and more accurate diagnostic testing, tailored medication, and positive performance. ML analyses patient's health and recommends critical functions to be made to prevent illnesses.
- *Drug Discovery and Manufacturing*. Pharmaceutical research and processing in creating a new drug, research and development technologies such as bioinformatics as well as personalized medical science, offer assisting mostly in the discovery of medications for a variety of health conditions, while machine learning helps speed up the process of creating or producing a new medication, that can be a costly yet time-consuming procedure, for example, Insitro, these have merged the latest technology such as data science, machine learning, as well as other modern laboratory equipment to monitor as well as develop biological prototype models that address issues which they could not previously answer.
- *Medical Imaging*. Healthcare scanning detects microscopic errors within scanning images of patients, thus like a consequence, allowing clinicians to make an accurate identification. Microsoft's InnerEye project, InnerEye is one scientific study that employs machine learning and artificial intelligence to provide novel tools towards the systematic, statistical evaluation on 3-dimensional radiographic images. Using these images, research used machine learning to distinguish malignancies from the healthy tissue.
- *Personalized Medicine/Treatment*. Individualized medication/therapy. The objective is to extract ideas from huge volumes of data and then apply them to make patients healthier on a personal level. This information can recommend personalised components as well as identify illness probability. IBM invited Watson healthcare and Watson's project using machine learning techniques. This leads to the creation of intelligent devices for the patient's improving health. Watson reduced the amount of time clinicians spend making treatment options by presenting doctors with personalised therapy suggestions that include a review of the latest studies, medical supervision, and research experiments.
- *Smart Health Records*. Updating health data on a daily basis would be both time- taking as well as exhausting. Following the successful completion of such massive project, another sector in which machine learning has begun to save time, energy, and money is the maintenance of healthcare data. Ciox, a European digital healthcare enterprise, utilizes machine learning methods to improve health information administration and exchange. Its purpose is to enhance access to clinical digital information, automate the company's performance, plus increasing the effectiveness of health data.
- *Predicting Diseases*. Researchers gain exposure on large amounts of information gathered using observatories, Internet, online platforms, as well as other sources. ML solutions such as artificial neural networks assist with collaborating through this knowledge as well as detecting all kinds of simple illnesses for serious chronic deadly diseases. A study conducted by the University of Nottingham in the United Kingdom implemented a methodology that used machine learning and artificial intelligence to examine individual patient records to estimate which patients might have heart problems over the next ten years.

## 2. Related Work

On this topic, we have highlighted many papers from heart-related prediction studies. Having approaches for predicting whether or not an individual may suffer from cardiovascular disease could be extremely valuable and beneficial for both the medical industry and individuals. While we are conscious of the risks associated with heart disease, we can raise public awareness and encourage people to take preventative action. As a result, numerous researchers have discovered various methods and models for spotting cardiac illness; the work below is the most recent in this area. Haq et al. [18] integrated several feature selection techniques with various classifiers. Data pretreatment was carried out by removing missing data and employing standard and min-max scalars. Three feature selection methods were employed to choose essential characteristics. The minimum redundancy maximal relevance feature selection method detects significant characteristics and eliminates duplicates. The selection of relief features. The algorithm chooses characteristics based on the weights assigned to them. These algorithms use the least relative downsizing and choice, picking features by updating coefficients and eliminating characteristics whose values approach zero. Zhao et al. [19] in their work investigated the cardiac breakdown rates as pulses changed using temporal analysis, machine learning, as well as CNN models. To choose crucial features, three feature selection techniques were used. Levy et al. [20] proposed using machine learning techniques to calculate the percentage of cardiovascular risk in individuals with severe DCM over the course of a year. The ML model generated 32 healthcare information highlights, from which information gain chose key highlights that were closely associated with heart illness. This work focused on heart infections in people who were using prescription drugs.

Zhou et al. [21] showed continuous arrhythmia heartbeat identification; parallel delta modulations and rotated linear SVM are two of the techniques used in this treatment. Photonic crystals enable the recognition of fluorescence. Paragliola and Coronato [22] developed a model for predicting the likelihood of cardiac events in hypertensive individuals, with ECG data as input. A convolutional neural network and a long short-term memory network were coupled to build a hybrid model by the researchers. Time-series data were utilized to detect a rise in hypertension early on the individuals. Kim et al. [23] created a method to identify cardiac disease using a neural network. The feature sensitivity analysis was performed to evaluate features which are significantly more relevant during prediction. The most sensitive characteristics were the most useful ones. Following the identification of important features, connected features were discovered by evaluating the total difference in sensitivity of attributes in response to a change in the value of one aspect. If one feature's value has a bigger influence on the sensitivity of another value than the mean difference in responsiveness of all features, it implies two variables. Machine learning was applied to assess cardiovascular disease immunoassay biomarker tests. This research employs PCA, PLSR statistical techniques, and advanced machine learning algorithms. Alizadehsani et al. [24] recognized machine learning for coronary artery disease, with datasets analyzed, weights researched, implementation approaches, and machine learning (ML) as the main strategies split down. Machine learning classifiers were employed in this investigation. All of the classification models tested prior to the hepatitis inquiry were beaten by the random forest classifier. Pahwa et al. [25] used a hybrid approach called SVM-RFE, which reduced unnecessary data and eliminated duplication. Random forest and *Naïve* Bayes are also used to forecast heart disease after features are selected. For subset assessment, use correlation-based feature selection (CFS). To recognize dimensionality, researchers used a hybrid approach that combined the best-first-search and CFS subset assessment methods. A model that employs or modifies the random forest approach for the prediction of heart disease, random forest is presented, and it outperforms the usual random forest technique.

In the study by Anderson et al. [26], the formulas for many heart disease outcomes, which are dependent on the measure of many traditional risk factors, were suggested. The cardiovascular risk prediction models was constructed by taking into account infarction, coronary heart diseases (CHDs), and stroke. The equations demonstrated a promising need to focus on and attempt to control different risk factors, like blood pressure, lipid levels, rising lipid, smoking, and glucose intolerance. In the study of Ahdal et al. [27], according to the “Asian phenotype,” Asian Indians appear to be more likely to develop cardiovascular disease, 2 diabetes types, and metabolic diseases (MetS). Various research studies have been conducted to investigate the link between MetS and insulin resistance (IR), in addition to an overabundance of iron. Serum ferritin (SF) levels are typically associated with IR measurements such as increased blood glucose and insulin levels.

Authors used a clustering technique to diagnose cardiac illness. In their model, correlation-based attribute subset selection was combined with such a search technique using *K*-means clustering. Verma et al. [11] discovered that incorporating multiple regression analysis into the proposed model obtained the highest results, including an accuracy of 88.40%. Aside from what has come before.

Hinchliffe et al. [12] used an unsupervised model-based clustering technique to assess cardiac involvement in systemic sclerosis. The data classification approach discovered some previously unknown links between the samples to forecast heart disease, and it advocated for recognize nonlinear classification algorithms. Bigdata methods, including HDFS and map reduction with the SVM, are recommended for use in forecasting heart disease because they detect an ideal set of attributes. The application of numerous data mining algorithms to detect heart disease was also investigated in this study. It is suggested that huge volumes of data be stored across numerous nodes using HDFS, and that the prediction algorithm be implemented using the SVM over multiple nodes at the same time. It is used in a similar way, returning a processing time that is quicker than standard time [28]. The data mining method when used with the ANN shows that for detecting heart illness, the expense of diagnosis has risen. New technology has been created to anticipate cardiac illnesses that are easily accessible and affordable. After analyzing the patient's health, the prediction technique is used to identify the patient's condition by recognizing several restrictions such as pulse rate, blood pressure, cholesterol, and so on. The framework is regarded as proper in Java. The provision of high-quality services at low prices is a major issue for healthcare institutions such as hospitals and medical centers. High-quality care involves appropriate patient diagnosis and appropriate therapy administration. The accessible heart disease database contains both quantitative and qualitative criteria. To eliminate any superfluous data from the database, these entries are cleaned and filtered before being submitted for subsequent processing [29, 30].

## 3. Research Methodology

Figure 3 shows various steps that have been taken in this study and are as follows:

- Loading the dataset
- Data loading is the procedure of copying and loading data or data sets from a source file, folder, or program into a database or related applications. It frequently involves capturing digitized data from a source, pasting it into a data storage or processing tool, and loading it 1.
- Data preprocessing

Preparing raw data for use is a step in the data mining process that involves preprocessing. Real-world data are frequently inaccurate, insufficient, inconsistent, or lacking in certain behaviours or trends. To solve such issues, a tried-and-true method is used for data preparation. Data preprocessing machine learning process steps are as follows:

**Step 1 .**

Import the libraries

**Step 2 .**

Load the dataset

**Step 3 .**

Look for any missing data

**Step 4 .**

Examine the categorical values

**Step 5 .**

Divide the dataset into two parts: training and testing

**Step 6 .**

Scaling the feature

- *Feature Selection*. The process of choosing the most important characteristics to feed into machine learning algorithms is known as feature selection, and it is one of the core elements of feature engineering. Feature selection procedures are used to reduce the number of input variables by deleting redundant or irrelevant features and narrowing the collection of features down to those that are most beneficial to the machine learning model. The primary advantages of performing feature selection in advance rather than letting the machine learning model determine which features are most important.
- *Feature Extraction*. It is a dimensionality reduction technique that compresses vast amounts of raw data into smaller bits for processing. Processing these big data sets needs a significant amount of computer resources due to the large number of variables. Feature extraction refers to techniques for selecting and/or combining variables to produce features, reducing the amount of data that must be processed while accurately and comprehensively describing the initial data set. Figure 3 displays the fundamental stages used for every machine learning models. Since relevant data cannot be analyzed immediately, data screening is first necessary. Significant features are then chosen, and these techniques are then applied to the prediction of each machine learning model.
- *ML Model*. In this case, a computational modeling “model” is the result of applying a machine learning algorithm to data. Deep learning system's findings are represented graphically by a model. The model, which contains the guidelines, figures, and other algorithm-specific data structures necessary to produce forecasts, is the “object” which is saved after a machine learning algorithm has been performed on training data.
- *Testing*. After a machine learning algorithm has been trained on an initial training data set, it is evaluated using a test set, which is a secondary (or tertiary) data set. Predictive models are supposed to always have some sort of unidentified potential that needs to be assessed rather than simply looked at from the perspective of programming.
- *Cross-Validation*. Is a statistical method for determining the capability of a machine learning model. Because it is simple to comprehend and use and produces skill estimates with less bias than some other approaches, it is commonly used in applied machine learning to compare and select a model for a specific prediction problem.
- *Result Prediction*. The term “prediction” refers to the output of an algorithm that has been applied to new data after being taught on old data to estimate the probability of a particular outcome, such as whether the patients have heart problems or not.

### 3.1. Dataset

The study was performed using a Cleveland heart disease dataset obtained from the UCI repository (University of California, Irvine). This dataset has 14 parameters 8 of which are categorical and 6 of which are numerical. The suggested methodology's flow is shown in Figure 3.

In Table 1, the properties and descriptions of the dataset are shown, and the dataset is summarized since there are 76 total characteristics, including the anticipated feature, and all research articles only implement a selection of 14 out of all. According to Estes' criterion, an electrocardiogram at rest with a value of 0 indicates probable or certain left ventricular hypertrophy. Thalassemia, ST, and major vessel size NULL for value 0 for slope peak exercise are already removed from the dataset. Value 1: fixed error (no blood flow in some part of the heart); blood flow is constant if the value is 2. Reversible value defect 3 is a blood flow that is observed but is not normal. If the patient has a heart problem, the “target” field indicates that it is an integer with a value of 0, representing no disease and 1, representing diseases. It is listed in Table 2 that there are 5 numerical and 9 categorical values, 1 duplicate row, and 0 missing elements.

In Table 2, data description, the number of variables is 14, and there are 303 observations, no missing values, only one duplicate row, and finally, there are two data types: 5 numeric and 9 categorical.

### 3.2. Classification and Regression Algorithms

*Classification*. It is a supervised learning approach that uses training data to recognize the nature of incoming observations. The classification algorithm analyses a certain dataset and then classifies new observations into one of several categories or groupings, for instance, yes or no, 0 or 1, and so on.

*Regression*. It is a sort of supervised learning in which the algorithm is trained with labels for both input and output. It helps to establish a relationship between variables by estimating how one variable impacts the other. There are different types of classification and regression using machine learning techniques:

#### 3.2.1. Logistic Regression

The logistic regression technique is considered one of the most suitable numerical models for estimating the probability of a particular class or event, such as success or failure [17]. The logistical regression employs numerous anticipated variables, which might be digital or class-based. This study also looked into the use of several data mining techniques to identify cardiac disease. Large amounts of data should be stored using HDFS across various nodes, and the prediction algorithm should be applied simultaneously across multiple nodes using the SVM. Similar to how it is employed, it provides a processing time that is faster than usual. A controlled machine learning method called logistical analysis is applied to “classified” issues. The logistics regression analyses the link among one or more separate characteristics to forecast the value of data based on previous observations of a data collection [31].

#### 3.2.2. Naive Bayesian (NB) Networks

A straightforward and efficient controlled learning method built on the Bayes theorem is the Naïve Bayesian algorithm. Less data are needed for training NB because it is based on likelihood and possibility. The existing class in NB is distinct from other classes, which is essential for categorization [32]. The *Naïve* Bayes technique simplifies predictive modeling and is typically used with large training datasets. Bayesian networks that are naive are incredibly clear. Bayesian network graphs with a single parent and a large number of offspring make up these networks. *Naïve* Bayes technique attempts to simplify the estimation problem by assuming that the unique input attributes, e.g., the different elements of the input vector, are conditionally independent. They are considered to be independent when they are not conditioned by the class, mathematically.

(1) $$\begin{array}{c} ANNs.p\left(\frac{c}{x}\right)=\frac{p\left(x/c\right)p\left(c\right)}{p\left(x\right)}\text{,} \end{array}$$

(2) $$\begin{array}{c} p\left(\frac{c}{x}\right)=p\left(\frac{x_{1}}{c}\right)p\left(\frac{x_{2}}{c}\right)*\ldots *P\left(\frac{x_{n}}{c}\right)p\left(c\right)\text{.} \end{array}$$

From equations (1) and (2), it shows that *P* (*c*|*x*), where *c* is the posterior probability of the target and *x* is the attribute predictor.

*P* (*c*) is the class prior probability. *P* (*x*|*c*) is the class likelihood offered by the predictor. *P* (*x*) is the predictor's prior probability.

#### 3.2.3. Random Forest

The Random forest method is one of the best methods for categorization and is able to sort huge volumes of data. It is employed for both regression analysis and classification. As the name suggests, the random forest approach is essentially made up of numerous separate decision trees that cooperate. An individual tree is distinct from all other trees with the same distribution. It is a supervised learning algorithm. It builds a “forest” out of DTs (decision trees). The “bagging” approach is frequently used to train DTs. This bagging strategy is based on the idea that by combining many learning models, the ultimate output may be improved. Although the difference was not substantial (particularly when compared to the difference in the patients' maximal heart rate), those who were well had a lower resting heart rate than those who were ill. On average, the difference was just 6 beats per minute. The advantage of this method is that it may be used for both classification and regression problems. The model becomes more random as the number of trees increases, thanks to RF (Random Forest). This strategy seeks the best feature from a random selection of characteristics to divide a node, rather than the best feature from a random selection of characteristics to split a node. This generates a diverse set of outputs, which typically improves the model's performance [33].

#### 3.2.4. KNN (K-Nearest Neighbors)

The k-nearest neighbor methodology is a straightforward yet effective classification technique. It makes no simplifying assumptions and is often used to solve classification problems when the data distribution is unknown. This technique employs the method of locating the *′k′* data points in the training set that are closest to the data point with the missing target value and applying the average value of the recovered data points to it. K-nearest neighbor is a classic machine learning methodology that employs supervised learning. The KNN approach assumes connection between both the fresh instance/input and previous cases then allocates the new case to the group closest similar to the original groups. This KNN approach keeps all previous data and utilizes similarity to categories' new data points. This implies that when raw data are generated, the KNN approach can swiftly categorize it into a suitable category. KNN does not make any assumptions about the underlying data because it is a nonparametric method.

From Figure 4, we assume we have two classes, *A* and *B*, and we have a new data point *k* = 1. This data point falls under which of the following classes? This kind of issue necessitates the use of the KNN technique. We can simply determine a dataset's category or class using KNN.

The Euclidean distance is defined as the distance between two points. It may be calculated as follows:

(3) $$\begin{array}{c} XandY:\surd \underset{1\leq i\leq n}{\sum }{\left(X_{i}-y_{i}\right)}^{2}\text{.} \end{array}$$

When the data have a large dimensionality, the Manhattan distance is frequently favored over the more common Euclidean distance:

(4) $$\begin{array}{c} \underset{1\leq i\leq n}{\sum }\left|X_{i}-y_{i}\right|\text{.} \end{array}$$

The Minkowski distance is defined as the distance between two variables:

(5) $$\begin{array}{c} {\left(\underset{1\leq i\leq n}{\sum }{\left|X_{i}-y_{i}\right|}^{p}\right)}^{1/p}\text{.} \end{array}$$

Here, *p* refers to a positive integer.

#### 3.2.5. Decision Trees

A flowchart or tree-like structure is used to illustrate the decision tree method. It uses a classification algorithm to address classification issues. Each branch represents a strong node value. The root node is completely surrounded by groups of instances. These instances are then sorted based on their features. In addition, it uses a decision tree-based ensemble machine learning approach with a gradient boosting framework. When employing high gradient boosting, two parameters require our attention. This approach selects the property with the greatest information gain after assessing sample homogeneity and information gain using entropy [32]. Decision trees (DT) classify occurrences by organizing them according to the value of their qualities. In a classification instance, each node of a decision tree represents a feature. Every branch indicates a positive node value. Instances are grouped all the way around the root node. The features of these instances are then used to sort them. Data mining and machine learning employ decision trees. In this strategy, a decision tree is employed as a prediction model. This model converts observations about an item into the goal value of the item.

(6) $$\begin{array}{c} Entropy\left(S\right)=\overset{c}{\underset{i=1}{\sum }}-p_{i}\log\;2p_{i}\text{.} \end{array}$$

Information Gain

(7) $$\begin{array}{c} Gain\left(S,A\right)=Entropy\left(S\right)-\underset{v\in values\left(A\right)}{\sum }\frac{\left.{\left|S\right.}_{v}\right|}{\left|S\right|}entropy\left(S_{v}\right)\text{.} \end{array}$$

#### 3.2.6. Extreme Gradient Boosting

Out of all the machine learning techniques, the extreme gradient boosting strategy is the quickest, most adaptable, accurate, and most versatile. A sort of ensemble machine learning technique called gradient boost is used to address problems in classification and regression-based predictive analysis. Tianqi Chen created it, and it is now part of the distributed machine learning community's larger set of open-source libraries. It is also a gradient boosting framework-based ensemble machine learning approach based on decision trees. We must pay attention to two parameters while using high gradient boosting. The first is gamma, which increases in value as the algorithm becomes more conservative. Subsample is the second parameter, and picking smaller values may help us avoid the problem of overfitting [33, 34].

## 4. Implementation and Result Analysis

To identify heart problems in patients, researchers used a variety of classification algorithms. Examples include decision tree, logistic regression, *Naïve* Bayes, random forest classifier, extreme gradient boost, and k-nearest neighbor. The Cleveland dataset from UCI was used in the tests. In Table 3, it shows that different columns and rows contain all values on the dataset, starting with age and ending with column 14th, which is the target column. Table 3 displays the head of the dataset by using data. Head () by default, it will show only the first 5 columns and rows.

In Table 4, we selected all of the numerical columns, took their average, and grouped them by our target column, “target” they are relatedly.

  data. group by (“target”)[[“thalach,” “chol,” “age,” “trestbps”]].mean()

Table 4 shows the average age of the individuals who presented with a cardiac ailment appeared to be 4 years younger than the people who arrived without a heart condition.

The maximum heart rates of sick and healthy people differ slightly. It is observed that healthy people have a 20 beats per minute higher maximum heart rate compared to average than sick people. Those who were not sick had a lower resting heart rate than those who were sick, though the difference was not significant (especially when compared to the difference in the patients' maximal heart rate) and only differed by 6 beats per minute on average. Finally, those who did not have heart disease had a lower cholesterol count of 8 mg/dL in their blood serum on average than those who did.

In Figure 5, it is the relation between blood cholesterol and age. The total cholesterol levels rise steadily from 20 to 65, then fall slightly in men and plateau in women. The elderly frequently have elevated cholesterol levels (61% of women aged 65 to 74). While remaining are a risk factor for coronary heart disease (CHD), elevated blood lipids become less noticeable over time after the age of 65, and their predictive value disappears by the age of 75, according to the graph.

In Figure 6, there is a small fudging (or grouping) to the right side of the plot for healthy persons, meaning that those who can attain greater maximum heart rates are more likely to have a healthy heart. It should also be noted that younger persons may attain greater heart rates per minute, showing that age and maximum heart rate have an inverse relationship.

In Figure 7, the direction of the slope on the peak of the ST (ST depression, oldpeak = ST depression caused by activity in comparison to rest) segment indicates the presence of exercise-induced angina. As a result, the typical ST segment during the activity has a much steeper slope.

Simply, for healthy people, the ST segment slope is predicted to ascend during effort testing.

### 4.1. Binning Continuous Numeric Values

Binning continuous features together and therefore creating discrete categorical columns could help the model generalize the data and reduce overfitting. I converted all the continuous values into categorical ones by binning them. The model is able to interpret the distributed weights of a particular feature when “there are fewer options to choose from” regarding observations.

  df = data
  df [“thalach”] = pd.cut (df [“thalach”], 8, labels = range (1, 9))
  df [“trestbps”] = pd.cut (df [“trestbps”], 5, labels = range (8, 13))
  df [“age”] = pd.cut (df [“age”], 12, labels = range (12, 24))
  df [“chol”] = pd.cut (df [“chol”], 10, labels = range (24, 34))
  df [“oldpeak”] = pd.cut (df [“oldpeak”], 5, labels = range (34, 39))

### 4.2. One-Hot Encoding Categorical Values

It is essential to encode the categorical features because, if not, the model may consider the numbers that represent categories as weights instead, which may result in the model identifying nonexistent correlations between the features. By specifying the drop first parameter to True, I used one-hot encoding with pandas.

### 4.3. Determining Feature Importance

We used a random forest classifier in order to determine feature importance and plotted them.

In Figure 8, we used a random forest classifier in order to determine important features, and then, we removed the remaining important features. This is a technique in which a score is assigned to each input characteristic for a certain model—the ratings simply indicate the “importance” of each element [35, 36]. A higher score indicates that the specific characteristic will have a greater effect on the model used to predict a certain variable.

### 4.4. Building the Model and Hyperparameter Tuning

 
*X* = *a*.drop ([“target,” “restecg_2,” “thalach_2,” “thalach_8,” “trestbps_12,” “age_13,” “age_22,” “age_23,” “chol_29,” “chol_30,” “chol_31,” “chol_32,” “chol_33,” “oldpeak_37,” “oldpeak_38”], axis = 1).
 
*Y* = data [“target”]
 
*X*_train, *X*_test, *y*_train, *y*_test = train_test_split (*X*, *y*, test_size = 0.20, stratify = *y*, random_state = 0)]

In order to decrease noise and overfitting, the target column and any feature columns with a significantly lower relevance percentage (such as the columns “chol 31” and “chol 32,” which were never utilized by the model to divide nodes) were removed. We utilized 80% of the data to train the model and 20% for testing, and we also used the stratification argument to ensure that both the training and validation sets had an equal number of persons who do and do not have heart disease. Finally, we utilized GridSearchCV to fine-tune hyperparameters while doing 10-fold cross validation.

Before implementing an algorithm, we should determine whether the data have been split evenly, as an uneven split will result in an issue with data balance.

  Print (*y*_test.unique ())
  Counter (*y*_train) [10].
  Counter ({0 : 110, 1 : 132})

## 5. Discussion

When compared to all other parameters combined, the use of ML on selected essential criteria produced the highest score in predicting heart disease, 96.72%. It is conceivable to conclude that the ML algorithm accurately predicts the risk of developing heart disease. The most prevalent qualities in healthy rules are sex = female, exang = no, and CA = zero (number of main vessels coloured by fluoroscopy). If a patient is female, no heart disease is predicted, no angina is provoked by activity, and no main arteries are coloured by fluoroscopy. Asymptomatic chest tightness is a key trait that appears in all diagnostic criteria for heart disease.

A positive relationship exists between a reversible thallium heart scan and an Oldpeak greater than zero. Males are more likely than females to develop heart disease since all of the bad rules indicated sex as male and all of the good rules stated sex as female.

In Table 5, different machine learning algorithms used in this paper are listed in Table 5. Whereas Table 6 shows the different result that are achieved by using ML algorithms. Then for evaluation, we used confusion matrix; it is a table which is widely utilized to explain the performance of the proposed model (or “classification algorithm”) on such a test data set under which the real data have been collected. It is the summary of prediction results. It helps us have a good data visualization.

From Table 6, we see that random forests have achieved the highest accuracy which is 96.72%, following extreme gradient boost with 95.08%, the lowest accuracy was obtained by decision tree 77.049%.

Table 7 shows the summary of all machine learning that has been used on this paper with their accuracy.

In Figure 9, the bar plot is showing the different machine learning techniques, and in Figure 9, random forest algorithm represent the highest accuracy followed by extreme gradient boost, and the lowest accuracy performed by decision tree which is 77.049%.

Using ML approaches, this section compares the proposed current works. The findings of this study show that the accuracy imposed on the random forest algorithm for 14 significant features has the highest score of 96.72% when compared to other latest research addressed in the literature study section that used the UCI Cleveland heart disease dataset in relation to the suggested proposal.

## 6. Conclusion

Heart diseases cause death globally, according to the World Health Organization, and the most common cause of death in heart disease is a delay in diagnosis. Machine learning technologies have made significant advances in disease detection. Many studies and records from many modern hospitals demonstrate the effectiveness of the ML technology. You could say that heart disease diagnosis and detection using machine learning algorithms are good predictors. The study's main contribution is the presentation of enhanced machine learning approaches for diagnosing heart diseases which are more accurate than existing methods. In this study, the Cleveland dataset UCI repository used, and the implementation was on Google Colab using Python language. Various machine learning algorithms have been used such as logistic regression 86.88%, *Naïve* Bayes 83.60%, random forest 96.72%, extreme gradient boost 95.08%, K-nearest neighbor 90.16%, and decision tree 77.049%. Random forest when compared to the previous work, it outperformed other machine learning algorithms mentioned in the literature section. It had the highest accuracy (96.7%). This research is not intended to replace the services of a doctor, but it could be useful in rural and remote areas in which there are no cardiac experts or other modern medical facilities. Furthermore, it may aid the doctor in making quick decisions. The recommended system has a number of drawbacks as well. It will only show us whether or not individuals have a heart condition. This method cannot determine the degree of heart disease.

## Figures and Tables

**Figure 1:** History of machine learning.

**Figure 2:** Machine learning applications.

**Figure 3:** Flow of the proposed methodology.

**Figure 4:** KNN algorithm.

**Figure 5:** Blood cholesterol.

**Figure 6:** Maximum heart rate.

**Figure 7:** Presence of exercises include angina.

**Figure 8:** Important features.

**Figure 9:** Bar plots represent the accuracy of ML models.

**Table 1:** Dataset values.

Original attribute name	New attribute name	Description
Age	Age	Age of the patient
Sex	Sex	Sex of the patient: 0 = female; 1 = male
Cp	Chest pain type	4 types of chest pain
Trestbps	Resting blood pressure	Resting blood pressure
Chol	Cholesterol	Serum cholesterol in mg/dl
Fbs	Fasting blood sugar	Fasting blood sugar > 120 mg/dl
Restecg	Resting electrocardiographic	Resting electrocardiographic results (values 0, 1, and 2)
Thalach	Maximum heart rate	Maximum heart rate
Exang	Exercise induced angina	Exercise induced angina
Oldpeak	ST depression	Oldpeak = ST depression caused by activity in comparison to rest
Slope	Slope peak exercise ST	Slope of the peak exercise ST segment
Ca	Number of major vessels	Number of major vessels (0–3) coloured by flourosopy
Thal	Thalassemia	Thal: 3 = normal; 6 = fixed defect; 7 = reversable defect

**Table 2:** Data description.

Overview	Values
Various variables	14
The quantity of observations	303
Absence of cells	0
Absence of cells (%)	0%
Identical rows	1
Identical rows (%)	0.30%
Total memory size	33.3 KiB
Average memory record size	112.4 B
Numeric	5
Categorical	9

**Table 3:** Data description.

No.	Age	Sex	Cp	Trestbps	Chol	Fbs	Restecg	Thalach	Exang	Oldpeak	Slope	Ca	Thal	Target
0	63	1	3	145	233	1	0	150	0	2.3	0	0	1	1
1	37	1	2	130	250	0	1	187	0	3.5	0	0	2	1
2	41	0	1	130	204	0	0	172	0	1.4	2	0	2	1
3	56	1	1	120	236	0	1	178	0	0.8	2	0	2	1
4	57	0	0	120	354	0	1	163	1	0.6	2	0	2	1

**Table 4:** Calculation of the average target.

Target	Thalach	Chol	Age	Trestbps
0	139.101449	251.086957	56.601449	134.398551
1	158.466667	242.230303	52.496970	129.303030

**Table 5:** ML techniques used for detection.

No	ML algorithm
1	Logistic regression
2	Naive bayes
3	Random forest classifier
4	Extreme gradient boost
5	K-nearest neighbour
6	Decision tree

**Table 6:** ML result compression.

ML algorithms	Confusion matrix	Accuracy (%)	Precision		Recall		*f*1-score		Support	
			0	1	0	1	0	1	0	1
Logistic regression	[[22 6] [2 31]]	86.88	0.92	0.84	0.79	0.94	0.86	0.89	28	33

Naïve Bayes	[[22 6] [4 29]]	83.60	0.85	0.83	0.79	0.88	0.81	0.85	28	33

Extreme gradient boost	[[25 3] [0 33]]	95.08	1.00	0.92	0.89	1.00	0.94	0.96	28	33

K-neighbors classifier	[[23 5] [1 32]]	90.16	0.96	0.86	0.82	0.97	0.88	0.91	28	33

Decision tree classifier	[[22 6] [8 25]]	77.049	0.73	0.81	0.79	0.76	0.76	0.78	28	33

Random forest	[[28 0] [2 31]]	96.72	0.93	1.00	1.00	0.94	0.97	0.97	28	33

**Table 7:** Summary of ML algorithm accuracy.

No	ML algorithm	Accuracy (%)
0	Logistic regression	86.885246
1	Naive Bayes	83.606557
2	Random forest	96.721311
3	Extreme gradient boost	95.081967
4	K-nearest neighbor	90.163934
5	Decision tree	77.049180

## Data Availability

The data used to support the findings of this study are available from the corresponding author upon request.
